# Effect and Safety Analysis of PRP and Yifu Combined with Ultrapulsed CO_2_ Lattice Laser in Patients with Sunken Acne Scar

**DOI:** 10.1155/2022/6803988

**Published:** 2022-01-25

**Authors:** Yuyan Wang, Wei Yu, Jufang Zhang, Jinsheng Li

**Affiliations:** ^1^Department of Plastic and Cosmetic Surgery, Affiliated Hangzhou First People's Hospital, Zhejiang University School of Medicine, Hangzhou 310006, Zhejiang, China; ^2^Department of Plastic and Cosmetic Surgery, Zhuji Hospital of Traditional Chinese Medicine, Shaoxing 311800, Zhejiang, China

## Abstract

**Objective:**

To investigate the effect and safety of PRP and Yifu combined with ultrapulsed CO_2_ lattice laser in patients with sunken acne scar.

**Methods:**

700 subjects were selected from the group of patients with sunken acne scar treated in our hospital from November 2010 to December 2020. They were divided into control group (*n* = 350) and study group (*n* = 350). The grouping was mainly based on the random number table method. Patients in the control group were treated with ultrapulse CO_2_ lattice laser, while those in the study group were treated with ultrapulse CO_2_ lattice laser combined with PRP and Yifu. The clinical effect, scar improvement and quality of life before and after treatment, and adverse events during treatment were compared between the two groups. The clinical effect was categorized into cure after treatment, significant effect, effective, and ineffective. The total effective rate = 1 − ineffective rate.

**Results:**

After treatment, the total effective rate of the study group (81.43%) was higher than that of the control group (70.00%). After treatment, ECCA, VSS scores, daily activities, symptoms and feelings, work and study, leisure and entertainment, interpersonal relationship, treatment status, and total scores were all lower in both groups than before treatment, and the study group was lower than the control group. During the treatment, the incidence of adverse events in the study group (17.33%) was lower than that in the control group (28.57%), *P* < 0.05.

**Conclusion:**

PRP and Yifu combined with ultrapulse CO_2_ lattice laser in the treatment of sunken acne scar can effectively improve the scar, reduce the incidence of adverse events, and the treatment effect is obvious, which can improve the quality of life of the patients.

## 1. Introduction

Acne is a chronic inflammatory skin disease that occurs on the sebaceous glands of hair follicles caused by a variety of causes. The main causes are related to abnormal hormone secretion, excessive sebaceous secretion, bacterial infection of propionibacterium acne, keratosis and blockage of hair follicle sebaceous ducts, and other factors. Women with endocrine system disorders and irregular menstruation and adolescent youths are at high risk [1, 2]. Acne is easy to relapse and aggravate repeatedly, resulting in complications such as pigmentation, persistent erythema, and sunken scar, among which sunken acne scar is more serious [3], mostly like orange peel, ice cone, meteorite crater, and so on. It greatly affects the normal life and mood of the patients [4, 5]. The treatment cycle of sunken acne scar is long. At present, in addition to drug therapy, physiotherapy is also increasingly used in the treatment of acne. Ultrapulsed CO_2_ lattice laser can accelerate the formation of keratinocytes, promote the proliferation and rearrangement of facial collagen and elastic fibers, and improve the symptoms of sunken scar, but the effect is slow when used alone [6]. Platelet-rich plasma (PRP) is a synergistic effect of a variety of growth factors released after platelet activation, which promotes the proliferation and differentiation of local repair cells and the synthesis of extracellular matrix, thus enhancing the ability of tissue regeneration and repair [7, 8]. At present, it has been widely used in clinical repair of chronic wound, bone and soft tissue injury [9–11]. Yifu is used to treat chronic skin ulcer wounds and burn wounds [12], in which the effective ingredient is recombinant human surface growth factor [13], which can accelerate the speed of cell wound repair [14]. The purpose of this study is to investigate the effect and safety of PRP and Yifu combined with ultrapulsed CO_2_ lattice laser on scar improvement in patients with sunken acne scar.

## 2. Materials and Methods

### 2.1. General Information

The basic data of the following two groups of patients was calculated and compared, suggesting that the difference in the data is not significant in the statistical study (*P* > 0.05), and then there was comparability between the two groups. 700 subjects were selected from the group of patients with sunken acne scar treated in our hospital from November 2010 to December 2020. They were divided into control group (*n* = 350) and study group (*n* = 350). The grouping was mainly based on the random number table method. The control group included the following: age 15–31 years, average 20.14 ± 2.07 years, 66 males and 84 females, and the course of disease ranged from 0.5 to 1.5 years, with an average of 0.98 ± 0.11 years. The study group included the following: age 16–32 years, mean 20.20 ± 2.11 years, 64 males and 86 females, and the course of disease ranged from 1 to 2 years, with an average of 1.09 ± 0.08 years. Diagnostic criteria: the diagnostic criteria of sunken acne scar in the recommended guidelines for clinical treatment of keloid are used as a reference. Inclusion criteria: those who meet the diagnostic criteria; those diagnosed by microscopic examination; those diagnosed by sex hormone test; those with informed consent of patients, etc. Exclusion criteria: patients with hypertrophic scar, patients with multiple infectious diseases, mental disorders, etc. The Medical Ethics Committee of our hospital has approved the implementation of this study.

### 2.2. Method

The patients in the control group were smeared with the appropriate amount of compound lidocaine cream (Tongfang Pharmaceutical Group Co., Ltd., Chinese medicine standard H20063466, specification: lidocaine 25 mg ropivacaine 25 mg/g) and then received ultrapulsed CO_2_ lattice laser, using pulsed carbon dioxide laser therapy apparatus (Beijing Hongqiang Furei Technology Co., Ltd., national equipment injection 20163241822, model: 10600AH). The full coverage electroacupuncture mode was selected to adjust the parameters around the scar with the frequency of 4 Hz for lattice, 20 min/times, once every 15 days. In the study group, on the basis of the control group, 40 ml of autologous elbow venous blood was taken 2 hours before treatment, and PRP was extracted by density gradient centrifugation. After the completion of ultrapulse CO_2_ lattice laser treatment, the wound was evenly smeared with PRP for 3 times with an interval of 1 month. At the same time, apply Yifu on the whole face after the laser lattice (national medicine standard S20020112, specification: 100,000 IU, Guilin Huanowi Genome Pharmaceutical Co., Ltd.).

### 2.3. Observation Index

① Clinical effect (including the cure after treatment): sunken scar basically disappeared, flat; significant effect: most of sunken scar disappeared, flat; effective: sunken scar improved compared with before treatment, but still not improved; ineffective: sunken scar did not improve or even aggravated. According to the consensus on early treatment of scar (version 2020), the total effective rate = 1−ineffective. ② Improvement of scar (including the acne scar weight score (ECCA)) before and after treatment reflects the severity of the scar, and the total score is 100 points; the higher the score is, the more serious the scar is; the Vancouver scar scale (VSS) score reflects the scar recovery, and the total score is 10; the higher the score is the worse the recovery is. ③ Quality of life (Including dermatology quality of life index (DLQI)) before and after treatment is divided into daily activities, symptoms and feelings, work and study, leisure and entertainment, interpersonal relationships, and treatment; each score is 3; the total score is 18; the higher the score is, the lower the quality of life is. ④ Adverse events include the occurrence of erythema, edema, and pigmentation during treatment, and the incidence of adverse events = (erythema + edema + pigmentation) cases/total cases × 100%.

### 2.4. Statistical Method

Statistical analysis was carried out with SPSS26.0 software, the measurement data were expressed as mean ± standard deviation ($\bar{x}\pm S$), the frequency was expressed as percentage (%), and the counting data were tested by *χ*^2^ test. Continuous variables were compared using Student's *t*-test. *P* < 0.05 was regarded as statistically significant.

## 3. Result

### 3.1. Clinical Effect

After treatment, it was found that the total clinical effective rate of patients in the control group (70.00%) was significantly lower than that in the study group (81.43%). After calculation, *P* < 0.05, as detailed in Table 1.

### 3.2. Scar Improvement

Compared with those before treatment, the scores of ECCA and VSS in the two groups decreased after treatment, and those in the study group were lower than those in the control group (*P* < 0.05), as detailed in Table 2.

### 3.3. Quality of Life

After treatment, the daily activities, symptoms and feelings, work and study, leisure and entertainment, interpersonal relationship, treatment, and total score in the study group were lower than those in the control group (*P* < 0.05), as detailed in Table 3.

### 3.4. Adverse Reaction

During the treatment, the incidence of adverse reactions in the study group was 17.33%, which was lower than that in the control group (28.67%). It was calculated that *P* < 0.05, as detailed in Table 4.

## 4. Discussion

It is clinically believed that the pathogenesis of acne is complex and diverse [15], but it is mainly due to the high level of androgen in the patient's body, and the sebaceous gland is affected by too much androgen secretion, which increases the amount of sebum produced. When combined with exfoliated secretions from the epidermis, it will block pores, resulting in acne [16, 17]. Like greasy, high calorie eating habits, high ambient temperature, staying up late, and high pressure are all inducing factors of acne [18], the typical clinical symptoms of patients are blackhead, pimples, nodular pustules, and cysts [19]. Sunken acne scar is caused by severe acne, repeated attacks, and improper nursing during the inflammatory period, which not only affects the facial beauty of the patients. At the same time, it brings inconvenience to the normal social communication of the patients [20, 21]. Treatments are divided into general treatment, drug therapy, physiotherapy, and other treatments [22]. In physiotherapy, photodynamic therapy, red and blue light irradiation, and intense pulsed light have a certain effect on the elimination of acne red marks [23]. Ultrapulsed CO_2_ lattice laser uses a gas laser to emit array-like light beams through an electroacupuncture laser, which can form some tiny thermal injury areas on the skin, where keratinocytes can regenerate quickly and accelerate wound healing, but the curative effect is slow when used alone [24].

The essence of PRP is to separate platelet and plasma by centrifugation and add thrombin to form gel to promote wound healing [25]. The therapeutic mechanism is that platelets can release brain-derived neurotrophic factor, vascular endothelial growth factor, and other growth factors after activation [26, 27]. A large number of studies have proved that PRP can promote the regeneration of cartilage and bone tissue, as well as anti-inflammatory and antibacterial effects [28]. In recent years, it has been widely used in bone and soft tissue reconstruction surgery, plastic surgery, diabetic foot refractory ulcers, and chronic skin ulcers [29]. Yifu is a kind of recombinant human epidermal growth factor for external use. It is mainly derived from polypeptides in mammals and is mainly used in the treatment of wounds, residual wounds, and ulcerative wounds after skin burns. The effect and safety of recombinant human epidermal growth factor extracted from natural substances are basically the same as those secreted by human body, and there are no side effects. At the same time of improving the symptoms of sunken scar, it also has a certain impact on the quality of life of patients [30].

In the results of this study, the total effective rate of the study group after treatment was higher than that of the control group, and the DLQI score was lower than that of the control group, and during the treatment, the incidence of adverse reactions in the study group was also lower than that in the control group, indicating that PRP and Yifu combined with ultrapulse CO_2_ lattice laser can effectively improve the therapeutic effect of patients with sunken acne scar, reduce the occurrence of adverse reactions, and then improve the quality of life of patients. ECCA and VSS are often used to evaluate the degree of scar caused by various skin problems. Yifu can promote the synthesis of nucleic acid and hydroxyproline in the cells around the skin wound, and at the same time, it can participate in inducing epidermal cells to mature and differentiate into stem cells and carry out scar epithelial cell proliferation and granulation tissue differentiation and development, so as to improve the scar condition and restore wound leveling [31, 32]. In the results of this study, the scores of ECCA and VSS in the study group after treatment were lower than those in the control group, indicating that PRP and Yifu combined with ultrapulse CO_2_ lattice laser can improve the scar condition of patients with sunken acne scar and facilitate the recovery of the disease.

In summary, PRP and Yifu combined with ultrapulsed CO_2_ lattice laser can effectively improve the scar of patients with sunken acne scar, reduce the incidence of adverse reactions, and the treatment effect is obvious, which can improve the quality of life of the patients. However, this study did not analyze the impact of inflammatory response in patients, and a multisample size and multicenter in-depth study is needed.

## Figures and Tables

**Table 1:** Comparison of the clinical efficacy of the two groups (*n* (%)).

Groups	*n*	Cure	Significant effect	Effective	Invalid	Total effective
Control group	350	47 (13.43)	82 (23.43)	116 (33.14)	105 (30.00)	245 (70.00)
Study group	350	56 (16.00)	91 (26.00)	138 (39.43)	65 (18.57)	285 (81.43)
*χ* ^2^						5.232
*P*						<0.05

**Table 2:** Comparison of the improvement of scar between the two groups ($\bar{x}\pm s$, score**)**.

Groups	*n*	ECCA		VSS	
		Before treatment	After treatment	Before treatment	After treatment
Control group	350	89.12 ± 7.08	69.21 ± 3.15^*∗*^	8.41 ± 1.14	5.65 ± 2.86^*∗*^
Study group	350	89.83 ± 6.98	49.38 ± 2.69^*∗*^	8.39 ± 1.21	3.55 ± 1.72^*∗*^
*T*		0.875	8.631	0.147	7.707
*P*		>0.05	<0.05	>0.05	<0.05

*Note.* Compared with before treatment, ^*∗*^*P* < 0.05.

**Table 3:** Comparison of the scores of quality of life between the two groups ($\bar{x}\pm s$, score).

Groups	*n*	Daily activities		Symptoms and feelings		Work and study		Leisure and entertainment		Interpersonal relationship		Treatment condition		Total score	
		Before treatment	After treatment	Before treatment	After treatment	Before treatment	After treatment	Before treatment	After treatment	Before treatment	After treatment	Before treatment	After treatment	Before treatment	After treatment
Control group	350	2.23 ± 0.46	1.16 ± 0.24^*∗*^	2.48 ± 0.22	1.73 ± 0.19^*∗*^	2.49 ± 0.23	1.71 ± 0.18^*∗*^	1.64 ± 1.08	1.48 ± 0.55^*∗*^	2.44 ± 0.33	1.58 ± 0.38^*∗*^	2.17 ± 0.51	1.69 ± 0.46^*∗*^	13.27 ± 1.35	10.06 ± 0.51^*∗*^	
Study group	350	2.28 ± 0.39	0.51 ± 0.13^*∗*^	2.51 ± 0.26	1.30 ± 0.09^*∗*^	2.43 ± 0.19	1.08 ± 0.20^*∗*^	1.66 ± 1.10	0.79 ± 0.24^*∗*^	2.45 ± 0.40	1.03 ± 0.16^*∗*^	2.12 ± 0.49	0.59 ± 0.30^*∗*^	13.22 ± 1.33	8.63 ± 0.34^*∗*^
*T*		1.015	29.166	1.079	25.050	2.463	28.676	0.159	14.083	0.236	16.337	0.866	24.531	0.323	28.573
*P*		>0.05	<0.05	>0.05	<0.05	>0.05	<0.05	>0.05	<0.05	>0.05	<0.05	>0.05	<0.05	>0.05	<0.05

*Note.* Compared with before treatment, ^*∗*^*P* < 0.05.

**Table 4:** Comparison of the occurrence of adverse reactions between the two groups (*n* (%)).

Groups	*N*	Erythema	Edema	Pigmentation	Total occurrence
Control group	350	30 (8.57)	35 (10.00)	35 (10.00)	100 (28.57)
Study group	350	21 (6.00)	25 (7.33)	14 (4.00)	60 (17.33)
*χ* ^2^					5.439
*P*					<0.05

## Data Availability

The datasets used and/or analyzed during the current study are available from the corresponding author on reasonable request.
